# G-Protein Coupled Receptor 35 Induces Intervertebral Disc Degeneration by Mediating the Influx of Calcium Ions and Upregulating Reactive Oxygen Species

**DOI:** 10.1155/2022/5469220

**Published:** 2022-01-18

**Authors:** Zhe Chen, Yucheng Jiao, Ying Zhang, Qingfeng Wang, Wenjian Wu, Jiancheng Zheng, Jitian Li

**Affiliations:** ^1^Department of Orthopaedics, Ruijin Hospital, Shanghai Jiaotong University School of Medicine, Shanghai 200025, China; ^2^Henan Luoyang Orthopedic Hospital (Henan Provincial Orthopedic Hospital), Henan Provincial Orthopedic Institute, Henan University of Chinese Medicine, Zhengzhou 450000, China; ^3^Shanghai Key Laboratory for Prevention and Treatment of Bone and Joint Diseases with Integrated Chinese-Western Medicine, Shanghai Institute of Traumatology and Orthopedics, Ruijin Hospital, Shanghai Jiaotong University School of Medicine, Shanghai 200025, China

## Abstract

Intervertebral disc degeneration (IDD) is a chronic disease affecting millions of patients; however, its specific etiology is unknown. G protein-coupled receptors (GPRs) are a superfamily of integral membrane receptors in cells, and the receptors respond to a diverse range of stimuli and participate in multiple cellular activities. Here, using RNA-sequencing (RNA-seq) methods and immunohistochemistry, we revealed that G protein-coupled receptor 35 (GPR35) may have a relationship with IDD. Then, we demonstrated that the deletion of *GPR35* in nucleus pulposus cells (NPCs) with siRNA or in *Gpr35^−/−^* mice significantly alleviated IDD caused by senescence or mechanical stress, further validating the pathological role of *GPR35* in IDD. In addition, *GPR35* induced the influx of Ca^2+^ and upregulation of reactive oxygen species (ROS) under mechanical stress in NPCs, which we believe to be the mechanism of GPR35-induced IDD. Finally, GPR35 caused upregulation of ROS in NPCs under mechanical stress, while excessive ROS stimulated the NPCs to express more GPR35 with a significant dose or time response. The u-regulated GPR35 could sense mechanical stress to produce more ROS and perpetuate this harmful cycle. In summary, our study shows that GPR35 plays a critical role in mediating IDD via mediating the influx of calcium ions and upregulating ROS, which implies a strong potential advantage of GPR35 as a prevention and treatment target in IDD.

## 1. Introduction

Intervertebral disc degeneration (IDD) is a chronic disease that affects millions of people and can lead to acute or persistent lower back or leg pain, anxiety, and motor dysfunction [1, 2]. Epidemiological investigations showed that the incidence rate of IDD in middle-aged and aged men and women is 62.4% and 54.7%, respectively, and the follow-up rate of new IDD in healthy volunteers is as high as 31.6% and 44.7% [2, 3]. Therefore, understanding how to effectively deal with the challenge of IDD is an urgent need.

It has been suggested that many etiologies may contribute to IDD (e.g., axial or shear mechanical stress, gene diversity, biochemical factors, or low-virulence anaerobic bacterial infection) [1, 4]. These factors affect IDD alone or in combination, and the pathological mechanism may be complicated and diverse. For instance, cellular receptors respond to many stimuli, such as mechanical stress, reactive oxygen species (ROS), and lipopolysaccharide, to participate in IDD processes. Of the receptors, the role of G protein-coupled receptors (GPRs) in IDD has attracted increasing attention.

GPRs are a superfamily of integral membrane receptors in cells and are characterized by a seven-transmembrane (TM) *α*-helical region [5, 6]. GPRs participate in nearly every cellular signaling event and physiological process, comprising approximately 800 known subtypes [5, 6]. The receptors respond to a diverse range of stimuli (e.g., photons, lipids, carbohydrates, amines, small chemical mediators, and complex proteins [5, 6]) and even mechanical stress [7]. Given the important role of GPRs in cellular function, nearly 40% of all pharmacopeia target these receptors [5, 6].

However, there are no reports on the function of GPRs in intervertebral disc (IVD) disease. Through a screen of GPR genes in IDD using RNA-sequencing (RNA-seq) methods, we identified G protein-coupled receptor 35 (GPR35) as potentially associated with IDD. We hypothesized that GPR35 participates in the pathological process of IDD under mechanical stress or autosenescence. In addition, we hypothesized that excessive ROS expression and Ca^2+^ influx may contribute to GPR35-related IDD. This research on GPR35 facilitates the development of targeted drugs for the management of IDD.

## 2. Methods

### 2.1. Patients and Tissue Collection

The study was approved by the Institutional Review Board of Ruijin Hospital, Shanghai Jiaotong University School of Medicine, and each participant signed an informed consent form. The patients who underwent posterior lumbar discectomy at our hospital because of lumbar intervertebral disc degeneration were enrolled in this study between February 2021 and September 2021. The nucleus pulposus (NP) was obtained during surgery and stored for subsequent experiments.

### 2.2. Human Nucleus Pulposus Cell (NPCs) Extraction and Treatment

After being harvested from surgery, samples were digested and cultured as previously reported [8]. Before compression, NPCs at the 2^nd^ passage were harvested and mixed with Corning matrix gel (Cat No. 356234, Corning, USA) for three days. For compression treatment, we set compression of 20 kPa for a duration of 0, 2, 4, and 6 hours with a Flexcell FX-5000 Tension System. To induce age-degenerated NPCs, the cells in the next passage were cultured for an additional two days after transfection. For transfection, we mixed Lipo fectamine3000 (Cat No. L3000001, Thermo Fisher, USA) with specific siRNA: 5′-AGGAGCACCCGGCACAAUUUCTT-3′; 3′-GAAAUUGUGCCGGGUGCUCCUTT-5′ (Sangon Bioengineering (Shanghai) Co., Ltd., Shanghai, China).

### 2.3. Compression of Caudal Intervertebral Disc (IVD) in Mice

All animal experiments in this study were approved by the Animal Care and Use Committee of Shanghai Jiaotong University School of Medicine, and we followed the protocols of the National Institutes of Health Guide for the Care and Use of Laboratory Animals (NIH Publications No. 8023, revised 1978). To induce IDD, an Ilizarov-type compression apparatus (Shanghai Yeyu Biotech Inc., Shanghai, China) was placed to induce axial compression at the caudal 7-8 of mice. In brief, two cross 0.4 mm diameter wires were inserted percutaneously into each of the 7th and 8th caudal vertebrae. The two wires were perpendicular to each other and parallel to the endplates of vertebrae. Then, the two wires were attached to two specifically manufactured resin rings that were connected longitudinally with four threaded rods. Finally, axial loads were applied using calibrated springs installed over each rod, which were tightened from the distal side. A thin-film pressure sensor was placed between the springs and rings to detect the pressure produced by springs, and the force between each spring and the ring was measured by sensors and fixed at the same level. The pressure was measured daily and guaranteed at the initial strength via fixing of the springs. Axial compression pressure was fixed at 0.8 MPa with a duration of 0, 6, 12, and 24 hours. The GPR35^−/−^ mice were provided by Professor Wang Chuandong (Xinhua Hospital, Shanghai Jiaotong University School of Medicine).

### 2.4. Western Blot Analysis

Protein extraction was conducted with RIPA according to the manufacturer's instructions (Cat No. P0013B, Beyotime, Shanghai, China). After extraction, total proteins were separated by SDS-PAGE, transferred to PVDF membranes (0.45 *μ*m, Millipore, Bedford, MA, USA), and incubated with primary antibodies against human aggrecan (cat No. A11691, ABclonal, China), collagen II (Cat No. 1560, ABclonal, China), and GPR35 (Cat No. PA5-23237, Thermo Fisher, USA). After transferring protein to the membranes, the membranes were incubated with a horseradish peroxidase-conjugated secondary antibody, goat anti-rabbit IgG (Cat. No. 7074, Cell Signaling Technology, MA, USA), at room temperature for 2 h, and the bands were visualized using chemiluminescence (Millipore, Bedford, MA, USA). B-actin (Cat. No. BF0198, Affinity Biosciences Ltd., USA) served as the internal control. The images were analyzed using a Fusion FX7 (Vilber Lourmat, Marne-la-Vallée, France) and analyzed with ImageJ software.

### 2.5. Real-Time Quantitative PCR

RNA extraction and synthesis of cDNA were conducted using a specific kit of Takara Premix Taq (Cat no. R004A, Takara Bio Inc., Shiga, Japan) according to the manufacturer's instructions. An ABI 7500 Sequencing Detection System (Applied Biosystems, CA, USA) was employed for qRT-PCR detection and analysis using the SYBR Premix Ex Tag Kit (Cat no. RR420A, TakaRa, Shiga, Japan). The cycling conditions were set as follows: 40 cycles of denaturation at 95°C for 5 s and amplification at 60°C for 24 s. *GAPDH* served as a housekeeping gene, and all reactions were run in triplicate. The primer sequences (Sangon Biotech, Shanghai, China) used in this study were as follows:

human *GAPDH* forward 5′-CTTAGCACCCCTGGCCAAG-3′; reverse 5′-TGGTCATGAGTCCTTCCACG-3′; human *GPR35*: forward 5′-AGGGACAAGGGCAAGAGGACTG-′ reverse 5′-GCGGCAGGTGTCATCAAGGC-3′; human *COLLAGEN II*: forward 5′-GATAACAGTCTTGCCCCACTTA-3′; reverse 5′CAAGAACAGCATTGCCTATCTG-3′; human *AGGRECAN*: forward 5′-GATCCTTACCGTAAAGCCCATC-3′; reverse 5′CTCCAGTCTCATTCTCAACCTC-3′; human *MMP-3*: forward 5′-GGCAAGACAGCAAGGCATAGAGAC-3′; reverse 5′ACGCACAGCAACAGTAGGATTGG-3′.

Target gene expression was normalized to the expression of *GAPDH* using the 2^-△△Ct^ method. All data were then normalized to the average of the control group.

### 2.6. Histology and Immunohistochemistry (IHC)

For IHC analysis, nucleus pulposus (NP) tissue from humans was fixed with 4% paraformaldehyde for 24 h and then processed via routine paraffin embedding, sectioning, and deparaffinization. For the caudal IVDs of mice, the tissue was harvested and fixed with 4% paraformaldehyde for 24 h, then decalcified using 10% ethylenediaminetetraacetic acid (EDTA) for 1 month before routine paraffin embedding, sectioning, and deparaffinization. The sections were stained by a routine H-E and Safranin O-Fast Green Staining method. Subsequently, the sections were incubated with a rabbit polyclonal antibody GPCR 35 (Cat No. PA5-23237, Thermo Fisher, USA), collagen II (Cat No. GB11021, Servicebio, China), or aggrecan (cat No. GB11373, Servicebio, China) at 4°C overnight. A specific IHC kit (cat. No. K5007, Agilent DAKO Inc., CA, USA) was used for the process according to the manufacturer's protocol. Nuclei were counterstained with hemalum (cat. G1004, Servicebio Inc., Wuhan, China). The stained samples were observed and photographed under a microscope (Axio, Carl Zeiss, Oberkochen, Germany).

### 2.7. Flow Cytometric (FCM) Analysis

To measure ROS and influx of Ca^2+^ in NP cells, after digestion with cell recovery solution (Cat No.354253, Corning Inc, NY, USA), the NPCs were resuspended in a work solution of the ROS detection kit and Fluo-3 AM detection kit (cat. no. S0033S and S1056, Beyotime Biotechnology Inc., Shanghai, China). The incubation was performed for an additional 30 min at 37°C in the dark. After incubation, the NPCs were washed three times with PBS. Fluorescence was analyzed using MoFlo Astrios (Beckman Inc, CA, USA). We measured the mean fluorescence intensity (MFI) of FITC-A as a measure of relative ROS expression and Ca^2+^ influx.

### 2.8. Statistical Analysis

The data are expressed as the mean ± SD. We performed a two-sided Student's *t*-test for two-group analysis. Among three or more groups, one-way ANOVA with post hoc Tukey's HSD test was used. Two-way ANOVA with post hoc Tukey's HSD test was performed for repeated measurements. GraphPad Prism (version 8) was utilized for statistical analysis, and *P* < 0.05 was considered significantly different.

## 3. Results

### 3.1. Expression of GPR35 Is Correlated with IDD in Human

To reveal the role of GPR35 in IDD, we conducted RNA-seq in degenerated NPCs. To mimic the degeneration of NPCs, the cells were compressed with 20 kPa for 4 h and RT-PCR analysis revealed that the NPCs had remarkable degeneration under this condition (Figures 1(a) and 1(b)). As seen in the RNA-seq heat map of Figure 1(b), *GPR35* was significantly upregulated, suggesting it may have a correlation with IDD. To further validate the pathological role of GPR35 in IDD, we examined the expression of GPR35 in degenerated NP tissues from patients using IHC staining. As shown in Figure 1(c), there was a gradual increase of the GPR35 expression in NPs with higher degeneration levels, with a statistical significance. Collectively, these results indicate that the expression of GPR35 has a correlation with IDD.

### 3.2. Deficiency of *GPR35* Alleviates IDD in Aged Human NPCs and Mice

When NPCs are cultured for several passages, the cells undergo autosenescence. We thus knocked down the function of *GPR35* with siRNA in aged NPCs, and the results showed that the decreased gene expressions of main ECM, collagen II, and aggrecan were significantly rescued, while the increased gene expression of the catabolic factor of MMP-3 was significantly inhibited, as depicted in Figure 2. A similar result was seen in protein analysis, shown in Figure 2(b).

In addition to the in vitro study, we also examined the severity of IDD in aged *Gpr35*^−/−^ and wild-type mice at 14 months old. As shown in Figures 2(c) and 2(d), deficiency of *Gpr35* alleviated the severity of IDD as evidenced by a reduction of notochordal cell loss and fewer fissures in the annulus fibrosus, when compared with wild-type mice. IHC staining showed that the NPs of *Gpr35*^−/−^ mice reserved more collagen and proteoglycan than those of wild-type mice (Figures 2(e) and 2(f)). Taken together, these results indicate that GPR35 plays a critical role in medicating IDD in vivo and in vitro.

### 3.3. Inhibition of GPR35 Attenuates Mechanical Stress-Induced IDD In Vivo and In Vitro

After perceiving that deficiency of GPR35 alleviated aged IDD, we next intended to investigate whether GPR35 was also the key factor in mechanical stress-induced IDD. As depicted in Figures 3(a) and 3(b), the expression of GPR35 was increased in a time-dependent manner when NPCs were compressed in vitro. Next, we established an IDD model in mice by loading the Ilizarov setting on the caudal IVD. A similar trend of upregulated GPR 35 was found in vivo as depicted in Figure 3(c).

NPCs had decreased expression of main ECM proteins and increased expression of the catabolic factor when they experienced mechanical stress. However, this effect was abruptly knocked down in *GPR35* with siRNA, as depicted in Figure 3(d). Histological results of H-E and IHC staining showed that loss of GPR35 attenuated IDD as evidenced by *Gpr35*^−/−^ mice showing less deformation of NP, fewer twists of AF, and more reserved ECM (Figures 3(e) and 3(f)). Taken together, the results above reveal that GPR35 plays a critical role in mediating mechanical stress-inducing IDD in vivo and in vitro.

### 3.4. GPR35 Induces the Influx of Ca^2+^ and Upregulation of ROS under Mechanical Stress

Inhibition of GPR35-attenuated mechanical stress-induced IDD in vivo and in vitro; however, the mechanism remained unclear. Previous studies suggested that mechanical stress can induce upregulation of ROS in cells; therefore, we investigated whether GPR35 participated in mechanical stress-induced ROS. As depicted in Figure 4(a), along with an increase in compression, the level of ROS significantly increased in NPCs in a time-dependent manner. However, inhibition of *GPR35* significantly reduced the expression of ROS induced by mechanical stress (Figure 4(b)), suggesting that GPR35 responds to mechanical stress through the production of ROS.

As depicted in Figures 4(b) and 4(c), FCM results showed that the influx of Ca^2+^ significantly increased in a time-dependent manner, while the effect was inhibited when *GPR35* was knocked down using siRNA under mechanical compression. Consistently, activation of GPR35 induced by zaprinst significantly induced the influx of Ca^2+^ in NPC. Collectively, we believe that GPR35 induced the influx of Ca^2+^ and upregulated ROS under mechanical stress.

### 3.5. ROS Causes a Positive Feedback Loop of GPR35 Upregulation

It has been shown that a relationship exists between ROS and G-coupled receptor protein, and we have demonstrated that GPR35 causes upregulation of ROS in NPCs under mechanical stress. Interestingly, there have been previous studies on ROS-stimulated GPR overexpression. Therefore, we hypothesized that excessive ROS causes the upregulation of GPR35 and induces a positive feedback loop to deteriorate IDD. As depicted in Figures 5(a)–5(c), with an increase in H_2_O_2_ concentration or time exposure, GPR35 significantly increased in human NPCs, as demonstrated by gene or protein analysis, respectively. By contrast, when ROS that was caused by mechanical stress was neutralized by NAC, upregulated GPR35 was significantly decreased, as depicted in Figures 5(d) and 5(e). FCM showed that inhibition of GPR35 significantly reduced the influx of Ca^2+^ caused by H_2_O_2_ exposure in NPCs. Thus, we concluded that GPR35 caused upregulation of ROS in NPCs under mechanical stress, while excessive ROS caused positive feedback of GPR35 upregulation that led to IDD deterioration.

## 4. Discussion

In this study, we found that GPR35 plays a critical role in the process of IDD. Among the two most common pathogenic factors of mechanical stress and auto-senescence, inhibition of GPR35 function significantly alleviated IDD in vivo and in vitro. In addition, activation of the GPR35 with mechanical stress or agonist-induced Ca^2+^ influx and subsequent upregulation of ROS, which we considered as the pathological mechanism for IDD. Finally, we showed that mechanical stress can induce NPCs to produce excessive ROS via activating GPR35. The accumulated ROS subsequently induced upregulation of GRCP35 to sense more mechanical stress, which caused a harmful positive feedback loop to deteriorate IDD.

Of the GRCPs, GPR35 has gained significant attention because of its role in a broad range of diseases. For example, Zhang et al. suggested that the expression of GPR35 in bone marrow mesenchymal stem cells is suppressed in osteoporosis patients and osteoporotic mice, and that activation of GPR35 with agonist can rescue bone loss and promotes bone generation [9]. For cardiovascular disease, deletion of GPR35 induced augmentation of EC functions in vitro, enhanced endothelium-mediated vasodilation in isolated vessels, and prevented BP elevation *i*n vivo [10]. Activation of GPR35 can also protect against cerebral ischemia by recruiting monocyte-derived macrophages [11]. Therefore, regulation of GPR35 function with novel drugs has remarkable therapeutic potential to prevent and treat various diseases.

We first report here the pathological and pathophysiological role of GPR35 in IVD and IDD. In the aging model, deletion of GPR35 in mice significantly postponed the senescence of IVD, as depicted in Figure 2. Santos et al. determined that GPRs are potential platforms to control cellular senescence and consequently, age-related disorders [5]. The senescence of NPCs or IVD is complicated and the role GPR35 plays is also complex. During the aging process, the extracellular or intracellular repair system is impaired, and harmful stimuli, such as ROS, accumulate [12]. These stimuli may directly or indirectly activate GPR35 to induce degeneration of cells via different signaling pathways. In contrast, the senescence of NPCs is regulated by the aging paradigm, such as cell cycle arrest or dysfunction of cellular physiology [13], and GPR35 may affect the aging paradigm via cellular signaling networks [5]. Taken together, we believe that the deletion or deactivation of GPR35 with a drug or chemical compound is beneficial for IVD.

Aside from in vivo and in vitro aging models, we also tested the role of GPR35 in IVD under mechanical stress. Axial or shear mechanical stress is a well-known cause of IVD [14, 15]. Our data also suggested an increase of gradient pressure leads to the gradual degeneration of NPCs, as depicted in Figure 1(a). Previous studies reported that GPR, like G-protein-coupled receptor 68 [16], can sense mechanical stimuli. How GPR35 sense and transduce mechanical stimulation is unclear. Change of protein conformation under mechanical stimulation may result in subsequent cellular activity, or the G-protein-coupled receptor is regulated by other mechanical stimulation-related factors. Nevertheless, our data suggest that GPR35 plays a critical role in IDD caused by excessive mechanical stress, which is evidenced by data in vivo and in vitro.

The most plausible mechanism by which GPR35 induces IDD is causing the upregulation of ROS. The role of ROS in IDD has been verified in many studies [17, 18]. GPRs have always had a close relationship with ROS. It may induce the production of ROS via NF-kappaB activation [19] or directly regulate NAPDH oxidase [20]. Here, we also suggested that activation of GPR35 resulted in the influx of calcium in NPCs. The subunit of GPRs, activated G*α*, is able to interact and regulate many effector molecules such as potassium channels, adenylyl cyclase, phospholipase C (PLC), PLD, and protein kinases [6]. The subunit of G*βγ* also regulates adenylyl cyclase, phospholipase C-*β* (PLC-*β*), phospholipase A2 (PLA2), phosphoinositide 3-kinase (PI3-kinase), and *β*-adrenergic receptor kinase, some of which induce calcium regulation [6, 21, 22]. Increased levels of calcium always trigger the production of ROS [23], and excessive ROS subsequently resulted in damage of NPCs or IVDs [17], which was thought to be one of the mechanisms of GPR35-induced IDD.

We also observed an interesting phenomenon in which GPR35 conducted a harmful positive feedback loop between mechanical stress and ROS. Increased ROS stimulated the NPCs to express GPR35 with a significant dose or time response, and the upregulated GPR35 could then sense mechanical stress to produce more ROS to perpetuate this harmful cycle. Thus, NAC, the scavenger of ROS, successfully abrogated the harmful positive feedback in the system, as depicted in Figure 5. Previous reports also elicited that ROS had effects on GPRs [24] and expression of GPRs is regulated by multiple factors [5]. Although the mechanism is unclear, ROS is involved in various cellular activities; so, there may be complex network regulation that causes excessive ROS levels to upregulate GPR35. It was suggested that several potential promoters and enhancers participated in expression of GPR35, such as GH02J240620, GH02J240603, GH02J240583, GH02J240596, and GH02J240023, and ROS may have relationship with those promoters and enhancers. And more studies were needed to investigate the potential relationship. Nevertheless, we made a rational conclusion that elimination of excessive ROS may provide a novel way to inhibit the GPR35-related IDD.

Nonetheless, we should note the shortcomings of this study. First, the results of ROS and calcium detection were mainly acquired via FCS, which requires further exploration. Moreover, whether a deficiency of GPR35 can inhibit inflammatory- or infection-induced IDD needs to be further explored. In addition, various channels, such as Piezo channels or transient receptor potential (TRPs) channels, also played critical roles in mechanical stress-induced cellular activities. In this study, we proved that GPRs also sense mechanical stress. Is there any relationship between GPRs and Piezo or TRPs under mechanical stress? Which channels or receptors played predominant roles under mechanical stress? More studies were needed in the further to investigate the problem. Finally, the types of cellular signaling pathways that ROS regulates for the increased expression of GPR35 are also worthy of further investigation.

## 5. Conclusion

In summary, our study revealed that GPR35 plays a critical role in mediating IDD via the influx of calcium ions and upregulation of ROS, which implies a strong potential advantage of GPR35 as a prevention and treatment target in IDD.

## Figures and Tables

**Figure 1:** Expression of GPR35 is correlated with IDD. (a) RT-PCR analysis suggests that NPCs have downregulation of Collagen II and upregulation of MMP-3 when compressed with 20 kPa for 4 h. (b) RNA-seq heat map suggests an upregulation of the GPR35 gene when NPCs are compressed at the above degenerative condition. (c) IHC staining suggests a gradual increase of GPR35 expression in human NPs along with higher degeneration levels. (The data are shown as the mean ± SD. ^∗∗^*P* < 0.01 for comparisons between two groups. One-way ANOVA and Tukey's multiple comparison test were used for statistical analysis).

**Figure 2:** Deficiency of GPR35 alleviates IDD in aged human NPCs and mice. (a). Deletion of GPR35 gene expression with siRNA in aged NPCs rescued the decreased expression of collagen II and aggrecan and inhibited increased expression of MMP-3. (b). Expression of collagen II and aggrecan proteins was rescued when GPR35 was inhibited. (c, d) In mice aged 14-months old, knockdown of GPR35 alleviated the severity of IDD, showing less loss of notochordal cells and fewer fissures in annulus fibrosus. According to modified Thompson grade for histological grading of intervertebral disc in H-E straining, it was grade 2 and grad 3 for *GPR35*^−/−^ mice and wild-type mice, respectively. (e, f) The NPs in *GPR35*^−/−^ mice reserved more collagen and proteoglycan than those in wild-type mice. (Data are shown as the mean ± SD. ^∗^*P* < 0.05, ^∗∗^*P* < 0.01, and ^∗∗^*P* < 0.001 for comparisons between two groups. One-way ANOVA and Tukey's multiple comparison test were used for statistical analysis).

**Figure 3:** Inhibition of GPR35 attenuates mechanical stress-induced IDD in vivo and in vitro. (a, b) Overexpression of the GPR35 gene in a time-dependent manner when NPCs are compressed in vitro. (c) Increased GPCR 35 protein expression was found in caudal compressed IVD of mice. (d, e) Knocking down GPR35 with siRNA in NPCs rescued the mechanical stress-induced downregulation of main ECM proteins and upregulation of the catabolic factor. (f, g) Caudal IVDs in mice were compressed with the Ilizarov setting, and IVDs in *GPR35*^−/−^ mice showed less degeneration and more reserved ECM. According to modified Thompson grade for histological grading of intervertebral disc in H-E straining, it was grade 3 and grad 4 for *GPR35^−/−^* mice and wild-type mice, respectively. (The data are shown as the mean ± SD. ^∗∗^*P* < 0.001 and ^∗∗∗^*P* < 0.0001 for comparisons between two groups. One-way ANOVA and Tukey's multiple comparison test were used for statistical analysis).

**Figure 4:** GPR35 induces influx of Ca^2+^ and upregulation of ROS under mechanical stress. (a) FCM of DCFH-DA for ROS suggests the level of ROS significantly increased in NPCs with increase of compression in a time-dependent manner. (b) Inhibition of GPR35 significantly reduced the expression of ROS induced by mechanical stress. (c) FCM results show that influx of Ca^2+^ significantly increased in a time-dependent manner under mechanical compression. (d) Influx of Ca^2+^ was inhibited when GPR35 was knocked down using siRNA. (e) Activation of GPR35 by zaprinst significantly induced the influx of Ca^2+^ in NPCs. (The data are shown as the mean ± SD. ^∗^*P* < 0.05, ^∗∗^*P* < 0.001, and ^∗∗∗^*P* < 0.0001 for comparisons between two groups. One-way ANOVA and Tukey's multiple comparison test were used for statistical analysis among three groups. Student's *t*-test was used for statistical analysis between two groups).

**Figure 5:** ROS causes a positive feedback loop of GPR35 upregulation. (a)–(c) With an increase in H_2_O_2_ concentration or time exposure, GPR35 significantly increased in human NPCs with gene or protein analysis. (d) When ROS that was caused by mechanical stress was neutralized by NAC, GPR35 significantly decreased with gene or protein analysis. (e) FCM shows that inhibition of GPR35 significantly reduced the influx of Ca^2+^ caused by H_2_O_2_ exposure in NPCs. (The data are shown as the mean ± SD. ^∗∗^*P* < 0.001 and ^∗∗∗^*P* < 0.0001 for comparisons between two groups. One-way ANOVA and Tukey's multiple comparison test were used for statistical analysis among three groups).

## Data Availability

The data that support the findings of this study are available from the corresponding author upon reasonable request.

## Abbreviations

GPR35: G-protein coupled receptor 35
ROS: Reactive oxygen species
IVD: Intervertebral disc
IDD: Intervertebral disc degeneration
NPCs: Nucleus pulposus cells
NP: Nucleus pulposus.
